RETRACTED

# Meta-Analysis of the Comprehensive Efficacy of Intraocular Lens Implantation in Glaucoma Patients

**DOI:** 10.1155/2022/5130416

**Published:** 2022-08-16

**Authors:** Qingyi Zhou

**Affiliations:** Department of Ophthalmology. Zhejiang Provincial People's Hospital, People's Hospital of Hangzhou Medical College, 158 Shangtang Road, Hangzhou, 310014 Zhejiang, China

## Abstract

This study is aimed at investigating the efficacy of intraocular lens (IOL) implantation in patients suffering from glaucoma through meta-analysis of the previously published research. For this purpose, different literature databases were searched for identification of clinical studies published between January 2000 and January 2022 on evaluating IOL's efficacy in treating glaucoma. RevMan 5.3 was used to conduct a meta-analysis of the pertinent data. The central anterior chamber depth (ACD), corneal endothelial cell counts, best-corrected visual acuity (BCVA), intraocular pressure (IOP), anti-glaucoma medications (AGM), and axial length (AL) changes were compared, and the incidence of postoperative complications was thoroughly evaluated. The Cochran chi-square test was used to examine the heterogeneity of the evaluation results. According to the inclusion and exclusion criteria, 20 studies included 948 glaucomatous eyes. IOP was significantly lower than before treatment (MD = 8.64, 95 CI: 5.75-11.53; *Z* = 5.86, *P* < 0.0001), while ACD increased significantly (MD = −1.38, 95 percent CI: -1.74-1.02; *Z* = 7.49, *P* < 0.0001). The corneal endothelial cell counts were homogeneous (MD = 225.08, 95% CI: -64.17 to -514.33; *Z* = 1.53, *P* = 0.20). AGM utilisation decreased (MD = 1.43, 95% CI: 0.752.12, *Z* = 4.09, *P* < 0.0001). AL decreased significantly (MD = 0.31; 95% CI: 0.09-0.54; *Z* = 2.71; *P* = 0.007). The incidence of complications remained insignificant after IOL treatment (OR = 1.05, 95% CI: 0.42 to 2.60; *Z* = 0.10, *P* = 0.92; *P* = 0.92). These findings indicate that IOL treatment can significantly reduce intraocular pressure, glaucoma drug use, and aqueous level (AL) in glaucoma patients while increasing the depth of the central anterior chamber. This study offers a theoretical foundation for selecting glaucoma treatment methods.

## 1. Introduction

Glaucoma is a group of optic neuropathies characterized by structural changes in the optic nerve's characteristic head. In extreme cases, glaucoma can cause visual field loss and even blindness and is considered the second most common cause of blindness after cataracts. Glaucoma patients have increased in recent years due to people's growing reliance on electronic products and are a group of optic neuropathies characterized by structural changes in the optic nerve's characteristic head. The number of glaucoma patients worldwide exceeded 79.6 million in 2020, with more than 11 million suffering from binocular glaucoma. Approximately 10 percent of glaucoma patients are blind, accounting for more than 25 percent of all blindness cases [1]. China has a prevalence of glaucoma of 2.1%, which increases with age, and a blindness rate of 9.4% [2]. Damage to retinal ganglion cells and axons is the cause of glaucoma, which results in optic disc atrophy and changes to the visual field. Clinical glaucoma mainly includes primary glaucoma, congenital glaucoma, and secondary glaucoma. Primary open-angle glaucoma (POAG) and primary angle-closure glaucoma (PACG) are the two most prevalent types of glaucoma (PACG). Sixty to eighty percent of glaucoma cases involve PACG [3]. Primary angle-closure glaucoma was divided into three stages by the International Society of Geographical and Epidemiologic Ophthalmology: primary angle-closure suspect (PACS), primary angle-closure suspect (PACS), and PACG (ISGEO). Persistent or intermittent intraocular pressure elevations characterize glaucoma. The optic nerve of a patient with excessive intraocular pressure will become gradually atrophic, and the tissues of various eyeball parts and visual function will be severely damaged and affected, resulting in the gradual narrowing of the patient's field of vision, visual impairment, and eventual loss of visual ability [4]. When POAG and PACG are left untreated, the disease course is typically chronic, with progressive and irreversible visual field loss, which may result in tunnel vision and central vision loss [5]. To reduce the harm caused by glaucoma, early diagnosis, standard treatment, and reasonable evaluation of curative effects are crucial.

RETRACTED

The intraocular pressure lowering therapies have demonstrated their effectiveness in various randomized clinical trials [6]. Glaucoma is characterized by recurrence and difficult recovery following surgery. Due to issues with indications, mechanism of action, toxicity and side effects, and duration of drug therapy's efficacy [7], surgery is the most common clinical treatment. Currently, glaucoma filtration, intraocular lens implantation, cataract surgery combined with filtration alone, glaucoma surgery combined with cataract surgery, and glaucoma drainage implants are the most common surgical treatments for glaucoma. Glaucoma filtration is susceptible to complications, including shallow anterior chamber, cataract, malignant glaucoma, endophthalmitis, filter bubble leakage, and suprachoroidal hemorrhage [8]. Cataract surgery combined with filtration is effective, but it can speed up the formation of cataracts and cause functional follicles to vanish or shrink, limiting its clinical application. The combination of glaucoma and cataract surgery can significantly reduce intraocular pressure (IOP). Still, after surgery, the central visual field of patients is impaired, and several complications arise [9]. Intraocular lens implantation (IOL) releases the pupil block. It reopens all or a portion of the aqueous outflow channel for glaucoma, effectively reducing intraocular pressure and enhancing the patient's visual function when the channel is wholly or partially functional. The number of drugs used after IOL implantation is decreased, and some patients who have recovered well no longer require adjuvant drug therapy [10]. Biological ultrasound microscopy revealed that the thickness of the iris, ciliary body, and suspensory ligament did not change significantly after IOL implantation. However, the depth of the anterior chamber increased, indicating that the IOL replaced the eye's hypertrophic lens, and the iris regained its flat shape without contacting the IOL [11]. According to some studies, the IOP control rate was low in patients with glaucoma who were followed for nine months after IOL [12]. In addition, corneal edema, anterior chamber inflammation, posterior capsule rupture, retinal detachment, and other complications are possible following IOL surgery [13], and its safety requires further investigation.

There is still considerable controversy regarding the overall effectiveness of IOL in treating glaucoma. To explore the clinical effect of IOL in the treatment of glaucoma patients and to provide a reference for the treatment of clinical glaucoma patients, a meta-analysis was conducted on the therapeutic effect of IOL in the treatment of glaucoma at the national and international levels.

## 2. Materials and Methods

### 2.1. Data Inclusion Methods

For the study, glaucoma patients were chosen. Study types included randomized controlled trials (RCTs), prospective cohort studies, cross-sectional studies, and case-control studies. IOL surgery was the treatment administered to the participants. The data observations included the author, year, number of patients, number of eyes, duration of follow-up, patient's age, treatment methods, and observation indicators.

### 2.2. Literature Inclusion and Exclusion Criteria

The literature was subjected to prespecified inclusion and exclusion criteria for refinement. The inclusion criteria comprised of (i) articles published between January 2000 and January 2022 on IOL for glaucoma patients; (ii) the subjects which were more than one case of glaucoma patient who received IOL-related treatment; (iii) studies on the evaluation of the therapeutic effect of IOL for glaucoma patients, with detailed records of the therapeutic effect and indicators; (iv) the study types which were randomized controlled study (RCT), prospective cohort study, cross-sectional study, and case-control study; and (v) basic information which was recorded and central anterior chamber depth (ACD), corneal endothelial cell counts, best-corrected visual acuity (BCVA), intraocular pressure (IOP), antiglaucoma medications (AGM), axial length (AL) changes, and postoperative complication rate which were carefully recorded and statistically analyzed.

RETRACTED

The exclusion criteria are as follows: (i) individual case reports, literature reviews, expert comments, editorial opinions, news reports, product descriptions, and other publicity literature; (ii) literature without index data; (iii) literature lacking original data; (iv) repeated publications; (v) literature unrelated to the efficacy evaluation of IOL for glaucoma; (vi) literature that did not use IOL for treatment due to various reasons; and (vii) animal test, *in vitro* cell test, and other basic researches.

### 2.3. Retrieval Strategy

The retrieval time range for each online database was between Jan 2000 and Jan 2022. The search terms “intraocular lens (IOL) implantation,” “glaucoma,” “primary open-angle glaucoma (POAG),”“primary angle-closure glaucoma (PACG),”“treatment,” and “surgery” were entered into PubMed, Nature, Web of Science, Spring, and China National Knowledge Infrastructure (CNKI) by combining keywords with “or” and “and” from January 2000 to January 2022; published clinical studies on the efficacy evaluation of IOL in the treatment of glaucoma were searched by entering each keyword separately. The search was conducted without regard to language.

### 2.4. Selection of Literature and Evaluation of Quality

Two reviewers independently examined the quality of selected literature on the basis of the Cochrane Reviewer's handbook system. They extracted the data and excluded literature that did not meet the criteria or was of poor quality. In the event of inconsistent evaluation results, the reviewers involved were eligible to decide whether the literature was to be included or an opinion of a third reviewer was to be sought. All available variable information was extracted and entered into a Microsoft Excel database for the selected study.

The included literature was evaluated using the Cochrane Reviewer's handbook, version 5.1.0, by employing the following preset criteria: (i) correctness and preciseness of the research method, (ii) explanation of random sequence generation, (iii) clear and definitive research results, (iv) selectivity of reported results, (v) blind controlled study of participants and personnel in the article, (vi) results from an evaluation using the blind method, and (vii) data completeness and selective reporting. The included research was assessed according to the standard's seven criteria, with a total score of 7 points, and a score of 4 or higher was considered high-quality.

RETRACTED

The literature was reviewed initially based on the title, and missing information was collected by contacting the original author. After a careful reading of the abstract and entire text, the Jadad scale was applied to evaluate the quality of the contained literature. Inclusion in this meta-analysis was restricted to studies with a Jadad score greater than three.

### 2.5. Data Extraction

The included literature was extracted by two literature reviewers, with the literature extraction focusing on the following aspects: (a) basic information such as the title of the article, the first author, the publication year, the publication journal, the type of research, and the start and end dates of the study and (b) observation indicators: central anterior chamber depth (ACD), corneal endothelial cell counts, best-corrected visual acuity (BCVA), intraocular pressure (IOP), anti-glaucoma medications (AGM), axial length (AL), and postoperative complication rate.

## 3. Statistical Analysis

The data of the included literature was arranged using Microsoft excel 16, while Cochrane Reviewer's Handbook and Jadad scale were used to evaluate the quality of the literature. RevMan 5.3 was used for the meta-analysis of the included literature data.

The chi-square test was used for the preliminary heterogeneity test in the heterogeneity analysis, and the significance level was set to *α* = 0.05 and *P* < 0.05. Then, *I*^2^ in RevMan 5.3 was used to evaluate the heterogeneous results quantitatively. When *I*^2^ is less than 25%, heterogeneity in the literature is low. When 25% < *I*^2^ < 50%, moderate heterogeneity existed. When *I*^2^ > 50%, there was considerable heterogeneity in the literature. Based on this, the fixed-effects model was used for meta-analysis when *I*^2^ < 50%. When *I*^2^ > 50%, a random-effects model was used for meta-analysis. The measurement data are presented as the mean value (MD) and standard deviation (SD), and point estimates and confidence intervals (CI) for each effect size are provided. In describing dichotomous variables, relative risk (RR), odds ratio (OR), and risk difference were used (RD). RevMan 5.3 was used to generate a funnel plot to analyze publication bias. In the meantime, a forest map was developed, and the *Z* value and *P* value were extracted from the results to evaluate the meta-analysis results. The studies with the lowest quality scores were excluded from conducting sensitivity analysis. The inverted funnel plot was displayed as a funnel plot to observe publication bias in the literature. When *P* is less than 0.05, the difference between groups is statistically significant.

RETRACTED

## 4. Results

### 4.1. Literature Retrieval Process

After searching PubMed, Nature, Web of Science, Spring, China National Knowledge Infrastructure (CNKI), and Science Direct for “intraocular lens (IOL) implantation,” “glaucoma,” “primary open-angle glaucoma (POAG),” “primary angle-closure glaucoma (PACG),” “treatment,” and “surgery,” 1,023 articles were retrieved. Following an initial screening of duplicate literature, 165 relevant studies were included, among which 88 (PubMed), 40 (Web of Science), 20 (Spring), 12 (Nature), and five (Science Direct) articles were extracted. Sixty-seven studies were retrieved after removing those that did not fulfill the inclusion criteria; reviews, brief conference articles, case analyses, and risk factor evaluations were excluded based on the title, abstract, and substance of the literature. The initial screening identified 26 studies that met the inclusion criteria. After a thorough evaluation of the papers included in the study, six studies that we are unable to get original data were eliminated, leaving 20 studies for analysis (Figure 1).

### 4.2. Included Literature Basic Information

A total of 16 of the 20 references eventually included [14–33] provided data on the number of cases in the included studies, while 18 provided data on the proportion of female participants in the included studies. In the literature, 948 eyes with glaucoma treated with IOLs were included. The basic information of the literature included in this study is shown in Table 1.

### 4.3. Included Literature Quality Assessment

The Cochrane Reviewer's Handbook was utilized to assess the quality of the 20 included studies, and an evaluation chart was created to determine the overall quality of the literature. The results are depicted in Figures 2 and 3. Random sequence generation (selection bias), allocation concealment (selection bias), and blinding of participants and personnel (performance bias) were “low risk” in the 20 included studies. In two studies, blinding of outcome assessment (detection bias) was “high risk.” Blinding of outcome assessment (detection bias) was “unclear risk” in three studies but “low risk” in others. Incomplete outcome data (attrition bias) posed “uncertain risk” for three studies, “high risk” for one, and “low risk” for the remaining studies. There were four “uncertain risk” articles with selective reporting (reporting bias), two “high risk” articles, and no “low risk” articles. Another bias was classified as “uncertain risk” in three studies and “low risk” in the remaining studies. Therefore, the Cochrane Reviewer's Handbook's literature quality evaluations were above a B.

RETRACTED

The Jadad scale was then used to assess the quality of the included literature, which indicated that all included studies had a value of >3; hence, sensitivity analysis was unnecessary.

### 4.4. Comparison of IO*P* Values of Glaucoma Patients before and after Treatment

In the 20 included studies, the IOP values of glaucoma patients before and after IOL treatment were analyzed statistically, and the IOP values of glaucoma patients before and after IOL treatment were meta-analyzed (Figure 4). The IOP values of patients before and after IOL treatment were highly heterogeneous (*I*^2^ = 99%, *P* < 0.0001). Then, a random-effects model was used for analysis, and the IOP value of glaucoma patients after IOL treatment was significantly lower than that before treatment (MD = 8.64, 95% CI: 5.75-11.53; *Z* = 5.90, *P* < 0.0001).

### 4.5. Comparison of ACD Values of Glaucoma Patients before and after Treatment

A meta-analysis was conducted on the ACD values of glaucoma patients before and after IOL treatment, as reported by eight of the 20 studies (Figure 5). There was substantial heterogeneity between ACD values before and after IOL therapy (*I*^2^ = 98%, *P* < 0.0001). The combined effect values were analyzed statistically using the random-effects model. The results demonstrated that the ACD value of glaucoma patients treated with IOLs increased significantly compared to the value before treatment (MD = −1.38, 95% CI: -1.74-1.02; *Z* = 7.4; *P* < 0.0001).

### 4.6. Corneal Endothelial Cell Counts before and after Treatment in Glaucoma Patients

Four of the twenty studies analyzed the changes in corneal endothelial cell counts in glaucoma patients before and after IOL treatment. The corneal endothelial cell count of glaucoma patients was meta-analyzed before and after treatment (Figure 6). Before and after IOL treatment, there was considerable heterogeneity in corneal endothelial cell counts (*I*^2^ = 72%, *P* = 0.01). For the statistical analysis of the combined effect values, a random-effects model was applied. Comparing corneal endothelial cell counts before and after IOL treatment, there was no significant heterogeneity (MD = 225.08, 95% CI: -64.17 to -514.33; *Z* = 1.53, *P* = 0.13).

### 4.7. Comparison of Best-Corrected Visual Acuity (BCVA) before and after Treatment in Glaucoma Patients

Five of the included studies reported the changes in BCVA values before and after IOL treatment in glaucoma patients. Before and after treatment, the BCVA values of glaucoma patients were subjected to meta-analysis (Figure 7). There was considerable heterogeneity between patients' BCVA values before and after IOL treatment (*I*^2^ = 100%, *P* < 0.0001). The combined effect values were analyzed statistically using the random-effects model. Comparing BCVA values before and after IOL treatment, there was no significant heterogeneity (MD = 0.92, 95% CI: -1.25-3.09; *Z* = 0.83, *P* = 0.41).

RETRACTED

### 4.8. Comparison of Antiglaucoma Medication (AGM) Usage for Glaucoma Patients before and after Treatment

Nine studies provided data on AGM use in glaucoma patients before and after IOL treatment. Before and after treatment, a meta-analysis was conducted on AGM use in glaucoma patients (Figure 8). There was substantial heterogeneity between AGM usage before and following IOL treatment (*I*^2^ = 96%, *P* < 0.0001). The combined effect values were analyzed statistically using the random-effects model. After IOL treatment, the use of AGM in patients with glaucoma was significantly reduced compared to before treatment, with considerable heterogeneity (MD = 1.43, 95% CI: 0.75 to 2.12; *Z* = 4.09, *P* < 0.0001).

### 4.9. Comparison of Axial Length (AL) Values of Patients with Glaucoma before and after Treatment

Three of the included studies reported the changes in AL values in glaucoma patients before and following IOL treatment. Changes in AL values of glaucoma patients before and after treatment were investigated using meta-analysis (Figure 9). There was no considerable heterogeneity between AL values before and after IOL treatment (*I*^2^ = 42%, *P* = 0.18). The combined effect values were analyzed using a fixed-effects model. The results demonstrated that the AL value of glaucoma patients treated with IOLs was significantly lower than that before treatment, albeit with considerable heterogeneity (MD = 0.31, 95% CI: 0.09-0.54; *Z* = 2.71, *P* = 0.007).

### 4.10. Analysis of the Complication Rate of Glaucoma Patients Treated with OL

Five of the included studies statistically analyzed the incidence of complications in glaucoma patients treated with IOLs. A meta-analysis of the incidence of posttreatment complications in glaucoma patients was conducted (Figure 10). The incidence of posttreatment complications were insignificant among the IOL-treated patients (*I*^2^ = 0%, *P* = 1.00). Similar insignificant results were obtained when the fixed-effects model was applied (OR = 1.05, 95% CI: 0.42 to 2.60; *Z* = 0.10; *P* = 0.92).

### 4.11. Analysis of Publication Bias

The publication bias of the included literature was analyzed using an inverted funnel plot, and the results are presented in Figures 11–15. Notably, the inverted funnel plot of efficacy evaluation indicators and complication incidence of glaucoma patients before and after IOL treatment was symmetric, as were the majority of the included studies. In the funnel plot of IOP value and ACD value evaluation, only a few studies did not fall into the inverted funnel plot. Before and after IOL treatment, the efficacy evaluation indices and complication rate of glaucoma patients were close to the central axis. Based on this information, it was determined that the publication bias of the included literature used to analyze the comprehensive efficacy evaluation of glaucoma patients after IOL treatment was low and satisfied the requirements.

RETRACTED

## 5. Discussion

The leading cause of irreversible blindness is glaucoma. Its pathological basis is the apoptosis and progressive degeneration of retinal ganglion cells and their axons. The incidence of blindness due to glaucoma was 28.6%, significantly higher than the incidence of blindness due to cataracts (14.3%) [34], and more than $748 million was spent annually on glaucoma-related medical consultations, examinations, and surgeries [35]. China had the highest incidence of glaucoma among middle-aged and older women over the age of 50 years [36]. The peripheral iris obstructed the trabecular mesh, permanent adhesion with the trabecular mesh occurred, and aqueous outflow was obstructed, leading to elevated intraocular pressure and glaucoma. According to the findings of the present study, the incidence of glaucoma is associated with age, gender, race, and geographic location, and its pathogenesis is related to an increase in lens thickness, pupil block caused by the forward position of the lens-iris diaphragm, iris hyperfold, and nonpupilary block. Normal individuals have a central anterior chamber depth of approximately 2.5-3 mm, whereas glaucoma patients have a central anterior chamber depth of about less than 2.4 mm and 1.8 mm on average. When the central anterior chamber depth (ACD) was ≤1.4 mm, glaucoma incidence gets 100%. The incidence of glaucoma was 77.8% at 1.6 mm [37]. The glaucoma patients included in this study were treated with IOL. The results demonstrated that the ACD value of patients with glaucoma increased significantly after IOL treatment compared to that before treatment, with a significant difference between the two (MD = −1.38, 95% CI: -1.74-1.02; *Z* = 7.49; *P* < 0.0001). After IOL treatment, the ACD value of glaucoma patients increased significantly. After replacing an ocular lens with a thickness of less than 1.0 mm with an IOL lens (thickness = 4.0 mm), the central anterior chamber depth (ACD) was deepened, and the atrial angle was increased.

RETRACTED

Traditional glaucoma treatments include iris resection and filtration surgery, which are frequently accompanied by accelerated cataract formation, a shallow anterior chamber, purpura marks on filtration vesicles, and inadequate intraocular pressure control. IOL has the advantages of simple operation, small incision, less tissue damage, rapid visual recovery, short operation time, and fewer complications compared to these other methods. Current findings indicate that IOL implantation can reduce intraocular pressure in patients with glaucoma [38]. This study's meta-analysis revealed that the intraocular pressure (IOP) of patients treated with intraocular lenses (IOLs) decreased significantly compared to that before treatment (MD = 8.64, 95% CI: 5.75-11.53; *Z* = 5.86, *P* < 0.0001). This supports the conclusion that IOL implantation can significantly lower IOP in glaucoma patients. After replacing the human lens with an IOL, the volume of the eye's contents may decrease, the depth of the central anterior chamber may increase, and the contact plane between the pupil margin and the lens may shift posteriorly. Furthermore, cytokines such as interleukin-1 and prostaglandin released from postoperative aqueous outflow can promote degradation of the extracellular matrix of the trabecular meshwork, increase aqueous outflow, and thus reduce IOP [39].

Corneal endothelial cells play a crucial role in maintaining corneal health and transparency and regulating water and electrolytes inside and outside the cornea. Normal corneal endothelial cells are hexagonal mosaics with approximately 500,000 cells, averaging 2,570 cells/mm^2^ [40]. Loss of corneal endothelial cells can be brought on by corneal injury and various surgical procedures. Bullae keratopathy occurs when there are 10 to 15% fewer corneal endothelial cells than normal [41]. The results demonstrated that there was no significant heterogeneity in corneal endothelial cell counts after IOL treatment compared to before treatment (MD = 225.08, 95% CI: -64.17 to -514.33; *Z* = 1.53, *P* = 0.13), indicating that the loss of corneal endothelial cells in glaucoma patients was not significant after IOL treatment, thereby decreasing the likelihood of bullae keratopathy.

After surgery, glaucoma patients must continue to take anti-glaucoma medications. Currently, pilocarpine, prostaglandin derivatives, carbonic anhydrase inhibitors, and hypertonic dehydrating agents are the most widely used antiglaucoma medications. Current research indicates that long-term use of antiglaucoma medications induces varying degrees of ocular surface damage, affecting the trabecular meshwork and other structures, resulting in or exacerbating ocular surface diseases. It has been observed that the number of antiglaucoma medications used decreases after IOL implantation [42]. The results demonstrated that the use of AGM in glaucoma patients after IOL treatment was significantly reduced compared to before treatment, albeit with considerable heterogeneity (MD = 1.43, 95% CI: 0.75–2.12; *Z* = 4.09, *P* < 0.0001). It showed that patients treated with IOL required less antiglaucoma medication, but this study included few studies and made no comparisons to other surgical procedures. Therefore, the reduction in anti-glaucoma drug dosage for IOL-treated patients must be verified further. The atrial angle of glaucoma patients is significantly opened after IOL treatment, and the outflow pathway of aqueous outflow is reconstructed, thereby reducing the incidence of postoperative complications, as indicated by several domestic studies [43]. There was no significant heterogeneity in complications among glaucoma patients treated with IOL (OR = 1.05, 95% CI: 0.42 to 2.60; *Z* = 0.10, *P* = 0.92), indicating that the incidence of complications was low after IOL treatment.

RETRACTED

## 6. Conclusion

In this study, a meta-analysis was conducted to evaluate the overall efficacy of intraocular lenses (IOL) for postglaucoma. The results demonstrated that after IOL treatment, the ACD value increased significantly, the IOP value, the use of antiglaucoma medications, and the AL value decreased significantly, and the incidence of complications was low. Nonetheless, there are still some flaws in this study. Since most studies are observational, comparing and analyzing the efficacy evaluation indicators with other treatments are impossible. Additional clinical trials will verify the efficacy difference between IOL treatment and other glaucoma treatments. In conclusion, IOL therapy significantly decreased intraocular pressure, glaucoma drug use, and AOA in glaucoma patients while increasing the depth of the central anterior chamber. This work provides a theoretical foundation for the selection of glaucoma treatment methods.

## Figures and Tables

**Figure 1:** Literature retrieval and screening process.

**Figure 2:** Included literature bias assessment.

**Figure 3:** Risk evaluation of bias in selected studies.

**Figure 4:** Comparison of IO*P* values in glaucoma patients before and after treatment. CI: confidence interval; SE: standard error.

**Figure 5:** Comparison of ACD values of glaucoma patients before and after treatment. CI: confidence interval; SE: standard error.

**Figure 6:** Comparison of corneal endothelial cell counts in glaucoma patients before and after treatment. CI: confidence interval; SE: standard error.

RETRACTED

**Figure 7:** Comparison of BCVA values in glaucoma patients before and after treatment. CI: confidence interval; SE: standard error.

**Figure 8:** Comparison of AGM usage in glaucoma patients before and after treatment. CI: confidence interval; SE: standard error.

**Figure 9:** Comparison of AL values in glaucoma patients before and after treatment. CI: confidence interval; SE: standard error

**Figure 10:** Analysis of postoperative complications in glaucoma patients. CI: confidence interval; SE: standard error.

**Figure 11:** Funnel plot of IOP value assessment of glaucoma patients treated with IOL.

**Figure 12:** Funnel plot for ACD assessment of glaucoma patients treated with IOL.

**Figure 13:** Funnel plot of corneal endothelial cell count assessment in glaucoma patients treated with IOL.

**Figure 14:** Funnel plot of AL evaluation in glaucoma patients treated with IOL. SE: standard error; OR: odds ratio.

**Figure 15:** Funnel plot for evaluating the complication rate after IOL treatment in glaucoma patients. SE: standard error; OR: odds ratio.

**Table 1:** Included literature basic information.

First author	Year	Case number	Age (years old)	Eye number	Male/female (number of eyes)	Follow-up time (months)
Astle [14]	2009	27	60.7 ± 9.2	37	24/13	48
Chang [15]	2013	10	59.6 ± 10.7	10	6/4	46.3 ± 21.3
Dawczynski [16]	2007	/	66.6 ± 16.8	20	5/15	/
Gazzard [17]	2004	49	67.1 ± 7.6	49	29/20	/
Hata [18]	2008	27	75.8 ± 7.2	27	3/24	9.3 ± 6.3
Hayashi [19]	2001	/	73.6 ± 7.6	150	55/95	12
He [20]	2021	36	70 ± 8.83	36	9/27	6
Kashiwagi [21]	2006	21	76.9 ± 6.2	28	12/16	8
Ki-I [22]	2013	85	66.2 ± 6.9	85	23/62	21.9 ± 11.1
Kubota [23]	2003	15	/	18	11/7	6
Lee [24]	2010	26	68.8 ± 8.8	26	13/13	/
Parihar JKS [25]	2018	26	37.6 ± 10.25	26	14/12	9.6 ± 3.2
Pohjalainen [26]	2000	/	59.6 ± 10.7	38	/	44.4
Poley [27]	2009	/	75.5 ± 8.9	124	/	54 ± 12.8
Rhiu [28]	2012	23	68.57 ± 12.08	23	9/14	/
Su [29]	2011	14	72.63 ± 3.72	16	5/11	/
Tetz [30]	2015	21	76.3 ± 8.4	21	6/15	36
Tow [31]	2001	55	67.9 ± 9.2	57	25/32	22 ± 5.6
Yagev [32]	2019	73	14.3 ± 9.2	124	64/60	/
Zhao [33]	2013	33	69.6 ± 7.7	33	12/21	8.9

## Data Availability

The datasets used and/or analyzed during the current study are available from the corresponding author on reasonable request.
